# Molecular Basis of GABA Hypofunction in Adolescent Schizophrenia-Like Animals

This article has been retracted.

**DOI:** 10.1155/2021/9983438

**Published:** 2021-04-15

**Authors:** Xiaodan Wang, Ying Hu, Wenxin Liu, Yuanyuan Ma, Xi Chen, Ting Xue, Donghong Cui

**Affiliations:** ^1^Shanghai Mental Health Center, Shanghai Jiao Tong University School of Medicine, Shanghai, China; ^2^Shanghai Key Laboratory of Psychotic Disorders, Shanghai, China; ^3^Department of Neurology & Institute of Neurology, Rui Jin Hospital, Shanghai Jiao Tong University School of Medicine, Shanghai, China; ^4^Shenzhi Department of the Fourth Affiliated Hospital of Xinjiang Medical University, Urumqi, China; ^5^College of Life Sciences, Shanghai Normal University, Shanghai, China; ^6^Brain Science and Technology Research Center, Shanghai Jiao Tong University, Shanghai, China

## Abstract

Schizophrenia is a neurodevelopmental disorder that NMDA receptor (NMDAR) hypofunction appears centrally involved. Schizophrenia typically emerges in adolescence or early adulthood. Electrophysiological and several neurochemical changes have linked the GABA deficits to abnormal behaviors induced by NMDAR hypofunction. However, few studies have systematically investigated the molecular basis of GABA deficits, especially during adolescence. To address this issue, we transiently administrated MK-801 to mice on PND 10, which exhibited schizophrenia-relevant deficits in adolescence. Slice recording showed reduced GABA transmission and PVI^+^ hypofunction, indicating GABAergic hypofunction. Cortical proteomic evaluation combined with analysis of single cell data from the Allen Brain showed that various metabolic processes were enriched in top ranks and differentially altered in excitatory neurons, GABAergic interneurons, and glial cells. Notably, the GABA-related amino acid metabolic process was disturbed in both astrocytes and interneurons, in which we found a downregulated set of GABA-related proteins (GAD65, SYNPR, DBI, GAT3, SN1, and CPT1A). They synergistically regulate GABA synthesis, release, reuptake, and replenishment. Their downregulation indicates impaired GABA cycle and homeostasis regulated by interneuron-astrocyte communication in adolescence. Our findings on molecular basis of GABA deficits could provide potential drug targets of GABAergic rescue for early prevention and intervention.

## 1. Introduction

Schizophrenia is a devastating disorder that disrupts multiple brain systems, ending in decade-long psychosis and social and cognition impairment [1]. Although considered as a neurodevelopmental disorder [2], the onset of psychotic symptoms typically emerge in adolescence or early adulthood [1]. Recent findings suggest that therapeutic interventions during adolescence, typically before the onset of symptoms, might prevent or ameliorate the development of illness [3]. As the prefrontal cortex (PFC) continues to mature through adolescence and it is closely related to schizophrenia [4], understanding how PFC disruption occurs during adolescence will reveal key pathological mechanisms of illness and help early prevention and intervention.

NMDA receptor (NMDAR) hypofunction plays a key role in the pathophysiology of schizophrenia [5, 6]. This hypothesis is supported by the observations that NMDAR antagonists such phencyclidine, MK-801, and ketamine can produce schizophrenia-like symptoms in healthy humans and exacerbate preexisting symptoms in schizophrenic patients [7]. Rodents, repeatedly treated with NMDAR antagonists [6], during neonatal periods, also recapitulate schizophrenia-related behaviors, including locomotor hyperactivity, impairment of spatial learning and memory, and decreased sensory gating [8].

NMDAR hypofunction-related abnormal behaviors have been linked to excitation-inhibition (E/I) imbalance regulated by GABA deficits [9]. GABA (Ƴ-aminobutyric acid) is the principal inhibitory neurotransmitter in CNS released by GABAergic interneurons [10]. Electrophysiological recordings of NMDAR antagonists reveal reduced presynaptic GABAergic transmission and disinhibition of pyramidal neurons [9, 11]. Rescue with GABA_A_ receptor could restore behavioral deficits [9]. In animals, repeated injection of NMDAR antagonists reduces the expression of parvalbumin [12]. Bidirectional manipulation of parvalbumin and GAD67 (regulating GABA synthesis) levels in the mice hippocampus could regulate their learning ability [13]. In addition, postmortem studies of schizophrenia have persistently documented lower levels of parvalbumin [14, 15] and GAD67 [16, 17] in parvalbumin-positive GABAergic interneurons (PVIs^+^), indicating deficits in GABAergic circuits. Although electrophysiological and several neurochemical changes implicate the GABAergic deficits by NMDAR hypofunction, in addition, current data indicate the importance of astrocytes in regulating the dynamic GABAergic-astrocyte communication [18], and few studies provide a panoramic view of the molecular basis of GABAergic deficits, especially during the adolescence.

To address this issue, we transiently administrated MK-801 to mice on PND 10. They exhibited schizophrenia-relevant behaviors in adolescence. Accordingly, electrophysiological recording of PFC revealed reduced GABA transmission and PVIs^+^ hypofunction. We performed cortical proteomic studies and combined analysis of single-cell sequencing data from the Allen Brain. Integrative analysis of omics revealed that metabolic processes were differentially altered in excitatory neurons, interneurons, and glial cells. Notably, a set of GABA-related proteins regulating GABA cycle, consisted of synthesis, release, reuptake and replenishment, were downregulated. Particularly, these proteins were exclusively dysregulated in interneurons and astrocytes, indicating the impaired GABAergic-astrocyte communication. We revealed the molecular basis of GABA deficits, providing a global view of how GABA dysfunction occurred during adolescence. Our results may provide insight into the pathophysiological mechanisms of schizophrenia.

## 2. Materials and Methods

### 2.1. Mice and MK-801 Administration

For all experiments, we used wild-type C57BL/6 J male mice. All animal experiments were approved by the Experimental Animal Committee of Shanghai Jiao Tong University. Housing conditions include a 12 h light/dark cycle, a humidity of 50 ± 5%, and a controlled temperature of 22–25°C in the Individual Ventilated Caging System (IVC, TECNIPLAST S.P.A.). Food and water were provided ad libitum. The day of birth was defined as PND 1. On PND 10, pups were received two intraperitoneal injections of saline or MK-801 (Sigma-Aldrich) at a dose of 0.5 mg/kg (i.e., 10 ml/kg) at 9 : 00 AM and 17 : 00 AM, respectively. Mice were weaned on PND 21 and housed in single-sex groups (four to five per cage).

### 2.2. Behavioral Tests

A battery of behavioral tests related to schizophrenia, including open field test, elevated plus maze test, nesting building, Barnes maze, and prepulse inhibition test, were conducted in adolescent mice (~PND 35). Before behavioral tests, mice were acclimatized in the testing room for 1 h, and tests were conducted during 9 : 00 AM and 4 : 00 PM. The details of behavioral methods are provided in the supplementary methods. Electrophysiological recording, proteomic analysis, western blot, and immunohistochemistry were also performed in adolescent mice.

### 2.3. Electrophysiological Recording

Coronal slices were prepared from the PFC in an ice-cold and oxygenated sucrose solution containing (in mM) 212 sucrose, 3 KCl, 26 NaHCO_3_, 1.25 NaH_2_PO_4_, 0.5 CaCl_2_, 7 MgSO_4_, and 10 D (+) glucose. Following an incubation period of 30 min, recordings were performed in the oxygenated artificial CSF (ACSF). Micropipettes (4-6 M*Ω*) were filled with an intracellular solution containing the following (in mM): 130 K^+^ gluconate, 10 HEPES, 5 KCl, 0.5 EGTA, 10 phosphocreatine, 4 ATP-Na, 0.3 GTP-Na and 2.5 MgCl_2_, pH 7.23, and osmolality 313 mOsm/kg. Whole-cell patch-clamp recordings were obtained from PVIs^+^ or pyramidal neurons in the II/III layer of the prelimbic region (PrL). To measure intrinsic excitability, current was injected in 25 pA steps from 0 pA to 800 pA. Action potential (AP) threshold and frequency were recorded. sIPSC and sEPSC recordings (holding potentials of –70 mV) were monitored in pyramidal neurons. For sIPSC recordings, ACSF containing 10 *μ*M NBQX and 50 *μ*M APV and a high Cl intracellular solution were used. For sEPSC recordings, ACSF containing 100 *μ*M Picrotoxin and K^+^ gluconate intracellular solution was used. Data were acquired with a PatchMaster (HEKA, Germany) instrument and analyzed using MiniAnalysis (Synaptosoft, NJ). Data were normalized to the average baseline response. Cells whose access resistance exceeded 25 M*Ω* and had an unstable resting membrane potential or aberrant spiking pattern were excluded from the analysis.

### 2.4. Sample Preparation for MS Analysis

The PFC was mechanically homogenized (Dremel, USA) in the strong RIPA lysis buffer. 100 *μ*g of proteins was denatured in UA buffer (8 M Urea in 50 mM NH_4_HCO_3_, pH 7.8), reduced with 5 mM TCEP (Tris(2-carboxyethyl)phosphine), and alkylated with 15 mM IAA (iodoacetamide) for 30 min in the dark. Proteins were precipitated with precooled acetone and digested at 37°C for 18 h with trypsin (Promega) at a concentration of 1 : 50 (w/w) in 50 mM NH_4_HCO_3_. After digestion, peptides were desalted using a Mono spin column (GL Science, Tokyo).

### 2.5. Nano-LC-MS/MS

300 ng of peptides was reconstituted in 0.1% formic acid (FA) and separated by nanoscale reversed-phase UPLC on a nanoAcquity UPLC system (Waters Corporation), equipped with a Symmetry C18 5 mm, 180 *μ*m × 20 mm trap column and an HSS T3 C18 1.8 mm, 75 *μ*m × 250 *μ*m analytical column (Waters Corporation). Injected peptides were separated over a 120 min gradient from 3-35% B at a flow rate of 300 nL/min. Solvent A consisted of 0.1% FA in H_2_O, and solvent B was 0.1% FA in acetonitrile. The mass spectrometric analysis was performed on a Synapt G2-Si quadrupole time-of-flight mass spectrometer (Waters Corporation) in UDMS^E^ (ultradefinition MS^E^) mode. Positive ions in a mass range of 50 to 2000 m/z were acquired at a resolution mode of 20000 FWHM (full width at half maximum). A frequency of 30 s lock mass correction of [Glu1]-fibrinopeptide B was delivered.

MS raw spectra processing was performed in Waters Progenesis QI (QIP, version 3.0.2) as described previously [19], searched against the UniProt mouse proteomic database (version 2020/06). Default parameters for peak picking and alignment algorithm were applied. Carbamidomethylation of cysteine and oxidation of methionine were specified as fixed and variable modifications, respectively. A single missed trypsin cleavage was allowed. FDR for protein identification was set at a 4% threshold. Only peptides with a minimum length of seven amino acids identified with a confidence score ≥ 4 and<20 ppm mass error were considered.

### 2.6. Proteomic Data Analysis

Data normalization on peptide levels was performed automatically in the QIP software. Proteins were quantified using the Top 3 method [20, 21]. Only proteins with at least one unique peptide were considered. Duplicated technical replicates were performed. Proteins whose intensities were outside the range of the mean ± 2 sigma of each group were defined as outliers and removed. *K*-nearest neighbor (k-NN) imputation was applied to impute the missing values. The samr *R* package [22] was used to identify differentially expressed proteins using the paired two class of samr with 1,000 permutations and an FDR threshold of 0.05 [23]. Proteins identified with at least two unique peptides and a fold change of ≥ |1.3| were defined as differentially expressed proteins. Biological function analysis and protein-protein interaction were performed in STRING (http://string-db.org/), and the latter was visualized with Cytoscape 3.6.1 [24]. The protein expression in each cortical cell type was downloaded from the mouse brain single-cell sequencing database (http://mousebrain.org) [25].

### 2.7. Western Blot

Proteins were separated by 10% SDS-PAGE gel and blotted with primary antibodies as follows: mouse anti-PV (1 : 1000, Sigma), mouse anti-GAD65 (1 : 500, Abcam), rabbit anti-GAD67 (1 : 1000, Cell Signaling Technology), and rabbit anti-*β*-actin (1 : 2000, Cell Signaling Technology). The secondary antibodies used included goat anti-rabbit IgG (1 : 10000, Sigma) and goat anti-mouse IgG (1 : 10000, Sigma).

### 2.8. Immunohistochemistry

Brains were dissected and fixed overnight in 4% PFA at 4°C before cryoprotection in 30% sucrose. Brains were sectioned coronally in 20 *μ*m slices using a freezing microtome (Leica). Sections between bregma 1.54 mm to 2.46 mm were collected for cell counting. The primary antibody was anti-PV antibody (1 : 500; Sigma).The secondary antibody was Alexa Fluor 488 donkey anti-mouse antibody (1 : 000; Jackson lab). PVIs^+^ in the PrL region, consistent with electrophysiological recording, were counted every sixth of sections.

### 2.9. Statistical Analysis

Student's *t*-test was used when comparing two groups. Two-way analysis of variance (ANOVA) followed by post hoc Tukey's multiple comparison was used to analyze two factors and multiple group comparisons. A repeated measures ANOVA determined statistical differences of cumulative distribution. Statistical significance was defined as *p* < 0.05.

## 3. Results

### 3.1. Transient Blockade of NMDARs on PND 10 Induces Schizophrenia-Like Behaviors in Adolescent Mice

PVIs^+^ have been documented with the most sensitivity to NMDAR inhibition, especially during development [26]. PND 10 is when (1) mice brain growth reaches its peak [27], (2) maturation of mice cortical parvalbumin immunoreactivity of PVIs^+^ appears [28], and (3) excitatory synapses and fast-spiking properties of PVIs^+^ present in two days [29]. Hence, we targeted PND 10 as the critical point to induce NMDAR hypofunction. Male pups received two consecutive injections of MK-801 at 8 h intervals on PND 10. Considering the short half-life of MK801 (~2 h) in the brain [30], to effectively induce abnormal behaviors by the transient blockade strategy, a high dosage of MK801 (0.5 mg/kg) was chosen [31–33]. In contrast, a low (0.05-0.1 mg/kg) or moderate (0.2-0.25 mg/kg) dosage is generally used in the chronic treatment of rodents [8]. A battery of behavioral tests related to schizophrenia were performed during their adolescent stages (from PND 35) [34] when schizophrenia typically emerges in humans [1] (Figure 1(a)).

MK-801 injection on PND 10 did not affect mice weight in adolescence (Figure S1a). The open field test showed that mice locomotion activity was not disturbed (Figure S1b-c). Schizophrenia may increase comorbidity with anxiety disorders. We found that MK-801-injected mice spent less time in open arms while had a higher closed arm duration (Figure 1(b)), suggesting elevated anxiety-related activity. Next, we performed a PPI test to measure sensorimotor gating, which is frequently reduced in schizophrenic patients [35]. We observed no significant difference in baseline amplitude for the startle response (Figure 1(c)). However, MK-801-treated mice showed a significantly decreased prepulse inhibition at 85 dB (Figure 1(d)), indicating impaired sensory gating. Nest building is a measure of cooperative or social activity for rodents [36], whose decrease could correspond to negative symptoms in schizophrenic patients [37]. We found MK-801-treated mice exhibited a significantly lower ability of nest building (Figure 1(e)), who failed to build fluffy nests and tended to scatter pieces of cotton across the cage floor (Figure 1(f)). Impaired long-term explicit or declarative memory [38, 39] is one of the cognitive impairments in schizophrenia, which could be measured by the Barnes maze in rodents [40]. MK-801-treated mice showed significantly longer latency in entering the escape chamber than control mice across the four blocks of daily training (Figure 1(g)). However, the time spent in exploring the target hole in the probe test was not different between the two groups (Figure S1e). These data suggest learning but not memory ability was impaired in adolescent mice. Collectively, these observations demonstrate that transient blockade of NMDARs on PND 10 could induce schizophrenia-like behaviors in mice's adolescence.

### 3.2. Schizophrenia-Relevant Reduced GABA Transmission and PVIs^+^ Hypofunction Induced in Adolescent Mice

GABA deficits, especially PVI^+^ dysfunction, have been linked to the illness pathology of schizophrenia [14, 15]. Electrophysiological recording of reduced GABA transmission has been observed in NMDAR antagonist animals. Accordingly, we observed a significantly decreased interevent interval distribution and mean frequency of sIPSCs in the pyramidal neurons of MK-801-treated mice in adolescence (Figures 2(a)–2(c)). However, we found no significant changes in the cumulative amplitude distribution and mean amplitude (Figure 2(d)) in these neurons. These observations suggest a decreased GABAergic inhibitory input to pyramidal neurons. We next investigated the physiological function of PVIs^+^ in the PrL region. Fast-spiking features were used to identify PVIs^+^. The firing frequency of PVIs^+^ in MK-801-treated mice experienced a significant decline with increasing current injections (Figures 2(e) and 2(f)). However, we found no difference in action potential (AP) threshold (Figure 2(g)). These data suggest decreased excitability of PVIs^+^. We found no decrease in the density of PVIs^+^ (Figure 2(h)) or parvalbumin expressing (Figure 2(i)) in the PrL region, suggesting that the decreased excitability is likely due to a functional deficit of the PVIs^+^ and not a reduction in their numbers.

PVI^+^ control the E-I balance of neural circuits, and their inhibition is likely to disinhibit the activity of pyramidal neurons. However, we found no difference in AP threshold or firing frequency of pyramidal neurons when comparing mice from both groups (Figures 2(j)–2(l)). Mean amplitude, frequency, and both cumulative distribution of sEPSC in pyramidal neurons were also not different between groups (Figures 2(m)–2(o)), indicating that the excitability of pyramidal neurons was unaffected in adolescence.

### 3.3. Altered Global Proteome of PFC in Adolescent Mice

Treatment with MK-801 on PND 10 results in abnormal behaviors and GABAergic hypofunction in adolescence, reminiscent of schizophrenia. We next investigated the molecular basis of GABAergic deficit by proteomic analysis of PFC (Figure 3(a)). We generated high-quality proteomic data with high technical (median coefficient of variance (CV) < 10% and *R*^2^ > 0.9, Figure S2a-c) and intersample reproducibility (median CV < 15%, Figure S2d). Of the 4833 proteins identified, 3222 had a CV of technical reproducibility < 20% across all samples, and they were used for subsequent analysis (Figure 3(b)). 119 of cortical proteins were differentially expressed (DEPs) (fold change > ∣1.3∣, adjusted *p* < 0.05) in MK-801-treated mice (Figures 3(c) and 3(d)). Notably, 77% of the DEPs were downregulated (92 down v*s*. 27 up, Figure 3(c)). Their top Gene Ontology (GO) functions involved in different aspects of metabolic processes (Figure 3(e)). In contrast, we did not find significantly enriched biological function (data not shown) for the upregulated proteins. These data indicated impaired metabolic processes in adolescence of MK-801-treated mice. Hence, we hypothesized the observed reduction of GABA transmission in our electrophysiological recording that might be associated with the impaired GABA-related metabolic processes.

### 3.4. Integrative Analysis of Proteomics and Single-Cell Sequencing Revealed that Metabolic Processes Were Differentially Affected Depending on Cell Types

GABA-related metabolic processes could be coregulated by different cell types. Hence, we mapped the DEPs with the mouse single-cell sequencing data (http://mousebrain.org) to examine the cell-type specific functional alteration. We downloaded the expressed value of DEPs in their cortical cell types. We used hierarchical clustering to classify the cell types that DEPs have their most expression. We found DEPs were mainly clustered into three cell types: excitatory neurons, interneurons, and glial cells (Figure 4(a)). These cells were involved in different aspects of metabolic and developmental processes (Figures 4(b) and 4(c), Figure S3a-b). Reduced level of GABA is the core feature of GABA hypofunction. GABA is the naturally occurred amino acid working as the inhibitory neurotransmitter in the brain. What is interesting is that we found proteins enriched in interneurons and astrocytes which were both significantly enriched in the amino acid metabolic process (Figures 4(b) and 4(c)). In addition, astrocytes were also involved in the ion transport, which could be associated with neurotransmission (Figure 4(c)). Therefore, we further analyzed the proteins involved in the metabolic processes of the two cells. Notably, we found six of them were associated with GABA signaling, including GAD65 (encoding glutamate decarboxylase 65), SYNPR (encoding synaptoporin), GAT3 (encoding sodium and chloride dependent GABA transporter 3), SN1 (encoding sodium coupled neutral amino acid transporter 3), DBI (encoding acyl-CoA binding protein), and CPT1A (encoding carnitine O-palmitoyltransferase 1) (Figure 4(d)). These proteins were either from astrocytes or interneurons and were all downregulated in MK-801-treated mice. These data suggest impaired GABA signaling regulated by astrocytes and interneurons in adolescence.

### 3.5. Downregulated GABAergic Networks Coregulated by Interneurons and Astrocytes

We further analyzed how these GABA signaling-related proteins could affect GABAergic hypofunction. We found that the expression of GAD65, SYNPR, GAT3, SN1, DBI, and CPT1A showed a significant correlation with each other (Figure 5(a)), indicating their interaction in the network. Hence, we explored all the GABA-related proteins in our proteomic data. We found GAD65, SYNPR, GAT3, SN1, DBI, and CPT1A interacted with other GABAergic network components, like GAD67, GAT1, VGAT, PVALB, and GLU (Figure 5(b)). However, these interacted components were not changed in the MK-801-treated mice (Figure 5(b)). GABA is synthesized from glutamate by glutamate decarboxylase (GAD), which exists in two isoforms, that is, GAD65 and GAD67. Both GAD 65 and 67 are expressed in GABAergic neurons. We validated the downregulated expression of GAD65 by western blot, consisted with our proteomics result. However, the expression of GAD67 was not changed in MK-801-treated mice (Figures 5(c) and 5(d)). SYNPR is also expressed in GABAergic neurons. SYNPR interacts with the SNARE core complex and is responsible for synaptic vesicle fusion to regulate GABA release [41]. In addition, DBI can act on astrocytes' mitochondria to stimulate neurosteroid biosynthesis, which may regulate GABA_A_R [42] activity. GAT3 is a GABA transporter found on astrocytes to reuptake GABA and inactive GABAergic signaling [43]. Interestingly, SN1 is also exclusively expressed in astrocytes. It is required to release glutamine from astrocytes and furnish GABAergic neurons with the primary neurotransmitter precursor for GABA synthesis [44]. In addition, GABA release is known to be decreased through CPT1A reduction [45]. Thus, downregulation of these proteins suggest an inhibited GABA cycling (synthesis, release, termination, and replenishment) coregulated by GABAergic neurons and astrocytes in adolescence, which could explain the molecular mechanism of GABAergic hypofunction (Figure 5(e)).

## 4. Discussion

Here, we established a transient blockade of NMDARs on PND 10, which was sufficient to induce schizophrenia-relevant deficits in adolescent mice, such as deficits in sensory gating and impaired social and learning ability. Mice in adolescence exhibited reduced GABA transmission and PVI^+^ hypofunction by electrophysiological recording, indicating GABAergic deficits, which is the pathological feature of schizophrenia and consistent with previous studies by NMDAR antagonists [9, 11]. We then presented a cortical proteomic evaluation and combined analysis of single-cell sequencing data. We globally identified the molecular basis of GABAergic deficits induced by NMDAR hypofunction in adolescence, which is few investigated previously. Such fundamental overview could provide potential drug targets of GABAergic rescue for prevention and intervention.

Comparing the chronic blockade of NDMARs by antagonists during the neonatal period of rodents, the strategy of transient blockade on PND 10 showed a comparable effect on inducing schizophrenia-relevant behaviors. PND 10 is a critical time for the physiological maturation of PVIs^+^ [29]. PVIs^+^ are the major population of cortical GABAergic neurons and delicately control the excitation/inhibition balance [46]. Functional and molecular impairment of PVIs^+^ is frequently observed in schizophrenia. PVIs^+^ are more sensitive to NMDAR hypofunction compared to the pyramidal neurons [47], especially during development [48], due in part to its more highly expressed NMDARs in this period than in adulthood [49]. Genetic NMDAR ablation in PVIs^+^ during neonatal period, instead of the adulthood of mice, confers schizophrenia-like phenotypes [48], supporting the sensitive window of PVIs^+^ to NMDAR hypofunction. Hence, it is possible that the transient blockade of NMDARs on PND 10 alters the orchestrated process of PVI^+^ maturation, contributing to subsequent abnormal behaviors. Our results suggest that NMDAR hypofunction, even a subtle one during the critical stage of neonatal development, could have adverse effects amplified in later life, emphasizing the importance of neonatal health care.

Our study found impaired excitability of PVIs^+^ in adolescence, but not their amount or their PV immunoreactivity. We suggest that the observed reduced GABA transmission could be associated with the reduced excitability of PVIs^+^. The inhibition of PVIs^+^ is likely to decrease the strength of inhibitory inputs onto pyramidal neurons [9, 11]; however, in our study, we found that the excitability of pyramidal neurons was not affected. It could be a compensatory strategy to prevent excessive excitation and cell injury. Yet, additional studies will be required to confirm these findings.

We found that 77% of alternated proteins were downregulated in adolescence by postnatal MK-801 treatment. Some of them (e.g., GLOT1, PLXAN2, and TUBB5) have previously been associated with schizophrenia [50–52]. We found downregulated proteins were mostly enriched in a series of metabolic processes, in which excitatory neurons, interneurons, astrocytes, and oligodendrocytes were differentially affected. Energy-related and amino acid processes were preferentially disturbed in interneurons and astrocytes. Organic substance and nitrogen metabolic process was affected in excitatory neurons and oligodendrocytes. These differences might be associated with the different functions of NMDARs on these cell types. Studies have shown that MK-801 could affect glycolysis-related proteins in oligodendrocytes, but much less in neurons and astrocytes [53].

Notably, we identified that multiple GABA-related proteins were significantly downregulated in adolescence, including GAD65, SYNPR, DBI, GAT3, SN1, and CPT1A. These molecular participate in the GABA cycle, consisted of GABA synthesis, release, reuptake, and replenishment, to maintain the proper GABA homeostasis. Our finding indicates the molecular basis of GABAergic deficit observed in our electrophysiological recording, which could be resulted from the impaired GABA homeostasis.

GABAergic neurotransmission is comprised of phasic and tonic inhibition. The former is regulated by the classical vesicular release of GABA confined to the synapses, while the tonic inhibition involves the GABA spillover from the synapses and activates extrasynaptic receptors. GAD65 is located explicitly in axon terminals and specially regulates the vesicular release of GABA for synaptic transmission [54]. Although the evenly distributed cytosol GAD67 produces ~90% of GABA in the brain for cell metabolism and neurotransmission, it has been revealed that GAD65 is crucial to maintain the synaptic GABA by conversion of astrocytic glutamine via glutamate [55], especially when extensive synaptic GABA is required during peak demand [56, 57], so as to fine tune the GABAergic synaptic function. In addition, GAD65 is important in maintenance of the tonic inhibition [58], which has been estimated to constitute a prominent part of GABAergic transmission [59]. Evidence has suggested the key roles of tonic inhibition in memory, cognition, and schizophrenia [60]. GAD65^−/−^ mice exhibited pronounced deficits in pre-pulse inhibition [61]. Although postmortem studies have consistently shown lower expression GAD67 in the dorsolateral prefrontal cortex of subjects with schizophrenia, in our study, we did not find its alternation as previously reported. We suggested that the deficits in GAD65, rather than GAD67, could be the developmental feature of schizophrenia.

Astrocytes wrap around the pre and postsynaptic elements of neurons and exert profound effect on neuronal networks [18]. Current data support astrocytes' significance in regulating the dynamic GABAergic-astrocyte communication. Astrocytes regulate GABAergic synapses' activity by modulating the synaptic GABA content via its high-affinity transporters for GABA clearance and providing the neurotransmitter precursor for synthesis. Our study found that these two processes could be diminished in adolescence by downregulation of GAT3 and SN1. In addition to astrocytic clearance, GABA could be cleared from the synapses by uptake into the presynaptic neurons via GABA transporter 1 (GAT1). However, we did not find the alternated expression of GAT1, indicating that the process of neuronal clearance was not disturbed in adolescence. What is more, we suggest GABA_A_R signaling in astrocytes could also be inhibited by downregulation of DBI. DBI selectively knockout mice has shown certain forms of impaired spatial learning and memory [62]. NMDARs express in a low abundance on astrocytes. Activation of NMDARs on astrocytes could generate intracellular calcium signaling. However, their roles in astrocyticneuronal interaction in neurotransmission are unclear. Only one study reported that ablation or blockade of NMDARs on the hippocampus promoted the presynaptic inhibitory tone on excitatory neurons [63]. Collectively, we suggest that the inhibitory network mutually regulated by GABAergic neurons and astrocytes is impaired in adolescence, which could be astrocytic NMDAR-dependent or independent.

## 5. Conclusion

This study showed that a transient blockade of NMDARs postnatally had chronic behavioral and GABA deficits in adolescence. Our results revealed a downregulated set of GABA-related molecular, which synergistically regulate the whole process of GABA cycle, including GABA synthesis, release, reuptake, and replenishment. Although there have been studies targeting on GABA or other targets in new drug developments, our findings provided a comprehensive view of GABA deficits during adolescence, which is few studied. In addition, molecular like SYNPR, SN1, and CPTA1 has not been well investigated as drug targets. Hence, our study provided more clues and could benefit drug development.

## Figures and Tables

**Figure 1:** Mice administrated with MK-801 on PND 10 showed schizophrenia-like behaviors in adolescence. (a) C57BL/6 male mice intraperitoneally received two consecutive injections of MK-801 (0.5 mg/kg) or saline on PND 10 with an interval of 8 h. Behavioral tests were performed from PND 35. (b) Time spends in the open (*p* < 0.001) and closed arms, *p* = 0.0069. (c) There was no significant difference in the baseline startle response amplitude between MK-801-treated and control groups, *p* = 0.4083. (d) Prepulse inhibition was significantly inhibited at 85 dB in MK-801-injected mice (*p* = 0.0334). (e) Nesting building score was significantly lower in MK-801-treated mice, *p* = 0.0154. (f) The nesting building image between MK-801-treated and control mice. (g) MK-801-treated mice showed longer latency in entering the escape chamber (*F*_(1, 112)_ = 6.109, *p* = 0.015, two-way ANOVA). Data were represented as mean ± SEM. *n* = 14 of saline and *n* = 16 of MK801. ^∗^*p* < 0.05, ^∗∗^*p* < 0.01, ^∗∗∗^*p* < 0.001. Student's *t*-test for two groups' comparison. Two-way ANOVA by post hoc Tukey's multiple comparison for two factors and two group analysis.

**Figure 2:** Electrophysiological recording of pyramidal neurons and PVIs^+^ in the mPFC in adolescence. (a) Schematic diagram of whole-cell patch-clamp of sIPSC obtained from pyramidal neurons in the PrL region of mPFC. Saline or MK-801-treated mice were sacrificed on ~PND 30 and subjected for electrophysiological recording. (b) Example traces of sIPSC in pyramidal neurons. (c) Cumulative probability and the average frequency of sIPSC (saline/MK801: *n* = 10/9 cells from 3/3 mice per group, ^∗^*p* = 0.0224). (d) Cumulative probability and average amplitude of sIPSC (saline/MK-801: *n* = 10/9 cells from 3/3 mice per group, *p* = 0.5741). (e) Example traces of PVIs^+^ response to depolarizing current steps. (f) Input-output curve showing the average firing rate of PVIs^+^ in response to a series of increasing current steps. PVIs^+^ in the MK-801 group fired at an overall higher rate (two-way repeated-measures ANOVA, saline/MK-801: *n* = 8/9 cells from 4/3 mice per group, ^∗^*p* = 0.0365). (g) Average action potential threshold of PVIs^+^ (Student's *t*-test: saline/MK-801: *n* = 8/9 cells from 4/3 mice per group, *p* = 0.7731). (h) Density of cells with PVIs^+^ immunoreactivity in the PrL region. Student's *t*-test: *n* = 8 for each group, *p* = 0.9477. (i) Western blot analysis of PV immunoreactivity: *n* = 6/5 for the saline/MK-801 group. Student's *t*-test, *p* = 0.7783. (j) Example traces of pyramidal neurons in response to depolarizing current steps. (k) Average action potential threshold of pyramidal neurons (saline/MK-801: *n* = 13/15 cells from 3/4 mice per group, *p* = 0.2118). (l) Input-output curve showing the average firing rate of pyramidal neurons in response to a series of increasing current steps (two-way repeated-measures ANOVA, saline/MK-801: *n* = 13/15 cells from 3/4 mice per group, *p* = 0.5589). (m) Example traces of sEPSC in pyramidal neurons. (n) Cumulative probability and the average amplitude of sEPSC (saline/MK801: *n* = 12/10 cells from 4/3 mice per group, *p* = 0.4242). (o) Cumulative probability and the average frequency of sEPSC (saline/MK-801: n = 12/10 cells from 4/3 mice per group, *p* = 0.4544). Data were represented as mean ± SEM, ^∗^*p* < 0.05. Student's *t*-test for two groups' comparison.

**Figure 3:** Overview of the altered proteome of PFC in adolescent mice by data-independent UDMS^E^ approach. (a) Schematic diagram of data-independent proteomic acquisition. Saline or MK-801-treated mice were sacrificed on ~PND 30. The PFC was dissected for trypsin digestion and a 120 min gradient LC-MS acquisition. Duplicate technical replicates were performed for each sample. *n* = 5 of the saline group and *n* = 6 of the MK801 group. (b) 4833 proteins were identified, and only 3222 of them that the CV value of technical replicates ≤ 20% across all samples were used for subsequent analysis. (c) Volcano plot of significantly expressed proteins, Fold change ≥ ∣1.3∣, adjusted *p* < 0.05. (d) Hierarchical clustering of significant proteins. Each square represents one sample. Red: upregulated. Blue: downregulated. Protein's intensity was scaled across all samples and displayed as *Z* score. (e) The top GO enrichment of biological function of all significant proteins. Circle size represents the protein numbers in each item. *p* value was adjusted by FDR correction.

**Figure 4:** Integrative analysis of proteomics and single-cell sequencing data of differentially expressed proteins in adolescent mice. (a) All of the differentially expressed proteins in PFC identified in proteomics analysis were mapped to the mouse brain single-cell sequencing database (http://mousebrain.org). We downloaded the expression value of each differentially expressed protein within its clustered cell types in the cortex. A total of 45 cellular subtypes were showed, consisted of five major cell types of excitatory neurons, inhibitory neurons, astrocytes, oligodendrocytes, and microglia. Hierarchical clustering of the expression of significant proteins in all cell types showed their prominent cellular location. Red: higher protein expression. Blue: lower protein expression. Protein's expression was scaled in a row and represented as *Z* score. Pie graphs on the right panel showed the number and percentage of downregulated proteins in each cell type. (b, c) Top GO enrichment of biological function of differentially expressed proteins in interneurons and astrocytes. Circle size represents the protein numbers in each item. (d) Heatmap of differentially expressed proteins involved in the metabolic processes in astrocytes and interneurons. Proteins associated with GABA signaling were from astrocytes and interneurons and downregulated after postnatal MK-801 injection. Each square represents one sample. Red: upregulated. Blue: downregulated. Protein's expression was scaled in a row and represented as *Z* score.

**Figure 5:** Protein network analysis of GABA neurotransmission. (a) Pearson correlation analysis of the expression of significant proteins involved in GABA neurotransmission. The number inside the circle represents the *R* value. (b) Network of proteins involved in GABA neurotransmission. Blue: downregulated proteins. Grey: proteins whose expression were not changed in this study by MS analysis. Circle size represents the value of the adjusted *p* value. The larger size indicated the smaller *p* value. The *p* value of blue circles was below 0.05; otherwise, they were above 0.05. The thickness of lines represents the combined score of edges. (c) Western blot validation of the GAD65 expression, *n* = 6 of each group, *p* = 0.0043. (d) Western blot validation of the GAD67 expression. *n* = 6 of each group, *p* = 0.7108. Data were represented as mean ± SEM. ^∗∗^*p* < 0.01. Student's *t*-test. (e) Schema depicting the contribution of downregulated proteins in GABA dysfunction. GAD65 and SYNPR are responsible for GABA synthesis and release, respectively. GAT3 reuptakes GABA in the synaptic cleft. DBI is the GAGB_A_ receptor. SN1 transports GABA-derived glutamine to GABAergic neurons for GABA replenishment.

## Data Availability

The data used to support the findings of this study are available from the corresponding author upon request.

## Supplementary Materials

Supplementary Materials Fig. S1 Mice administrated with MK-801 on PND 10 showed schizophrenia-like behaviors in adolescence. Figure S2: quality control of proteomic data. Figure S3: integrative analysis of proteomics and single-cell sequencing data of differentially expressed proteins in early-adolescent mice. Supplementary Methods Information: open field test, elevated plus maze test, prepulse inhibition test, nesting behavior test, and Barnes maze.
